# Melanocytes determine angiogenesis gene expression across human tissues

**DOI:** 10.1371/journal.pone.0251121

**Published:** 2021-05-13

**Authors:** Shirly Freilikhman, Marianna Halasi, Alal Eran, Irit Adini

**Affiliations:** 1 Department of Life Sciences, Ben Gurion University, Beersheva, Israel; 2 Department of Surgery, Harvard Medical School, The Center for Engineering in Medicine, Massachusetts General Hospital, Boston, Massachusetts, United States of America; 3 Computational Health Informatics Program, Boston Children’s Hospital, Boston, Massachusetts, United States of America; Medical College of Wisconsin, UNITED STATES

## Abstract

Several angiogenesis-dependent diseases, including age-related macular degeneration and infantile hemangioma, display differential prevalence among Black, as compared to White individuals. Although socioeconomic status and genetic architecture have been suggested as explaining these differences, we have recently shown that pigment production *per se* might be involved. For example, we have shown that the extracellular protein fibromodulin is a pro-angiogenic factor highly secreted by melanocytes in White but not Black individuals. Still, additional pigment-dependent angiogenic factors and their molecular mechanisms remain to be identified. Understanding the contribution of pigmentation to angiogenesis in health and disease is essential for precision medicine of angiogenesis-dependent diseases with racial disparity. Toward that goal, we compared the transcriptomes of Black and White individuals in three tissues with angiogenic activity, namely artery, whole blood, and skin. We identified several differentially expressed angiogenesis pathways, including artery morphogenesis, regulation of endothelial cell chemotaxis, and cellular response to vascular endothelial growth factor stimulus. We then demonstrated that the expression of key genes in these pathways is directly modulated by the degree of pigmentation. We further identified the precise pigment production pathway controlling the expression of these genes, namely melanocortin 1 receptor (MC1R) signaling. These results demonstrate pigment-mediated regulation of angiogenesis-related pathways and their driver genes across human tissues.

## Introduction

An enormous amount of epidemiological evidence supports a correlation between the prevalence of angiogenesis-related disease and skin color. For example, age-related macular degeneration (AMD) is 55% less common in Black Americans and 46% less common in Asian Americans than in White Americans [1]. Likewise, White individuals are 1.5-fold more likely to present with infantile hemangiomas than are Blacks [2]. Similarly, rosacea is 3.3- to 3.8-fold more common in White, as compared to Black individuals [3]. Yet, the molecular bases for the disparities in the prevalence of these and other angiogenesis-related disease between Black and White individuals remain largely unknown.

Although Black and White individuals possess similar numbers of melanocytes, significant differences have been reported in melanocyte structure and function, as well as the degree of pigment production [4]. In skin, pigment-producing melanocytes are located in the basal layer of the epidermis, specifically within the extracellular matrix (ECM) that provides structural and biochemical support to surrounding cells. Melanocytes are also found in the eye, the inner ear, the heart, and most connective tissues, such as bone and meninges [5–7]. In addition to producing pigment, melanocytes can also affect gene expression and related functions of other tissues via secreted proteins [8–11]. Recently, we described a new paradigm wherein melanocytes regulate angiogenesis via secretion of fibromodulin (FMOD), an ECM protein belonging to the small connective tissue proteoglycan family [11]. We found that low pigment-producing melanocytes, such as those found in White individuals, express high levels of FMOD, which, in turn, promotes angiogenesis. In contrast, highly pigmented melanocytes, such as those found in Black individuals, express low levels of FMOD, leading to reduced angiogenic capacity. We have previously shown that melanocyte-secreted FMOD promotes angiogenesis in the microenvironment, in part by inducing TGF-β1 secretion by endothelial cells [11]. However, these and other angiogenesis-related processes modulated by pigment levels remain to be discovered. Moreover, it is still not known which differences in angiogenesis-related gene expression seen between Black and White individuals can be attributed to differential pigment levels, as opposed, for example, to common genomic variation. Understanding pigment-dependent gene expression is, therefore, essential for elucidating the molecular mechanisms underlying angiogenesis-related diseases characterized by racial disparity, and ultimately adopting precision care approaches for their management.

In the present study, we compared the transcriptomes of Black and White individuals in three tissues with angiogenic activity, namely artery, whole blood, and skin. We identified several differentially expressed angiogenesis pathways, including artery morphogenesis, regulation of endothelial cell chemotaxis, and cellular response to vascular endothelial growth factor stimulus. We further demonstrated that pathway genes differentially expressed between Black and White individuals, including *VEGFA*, *APOE*, and *FGFR*, are expressed by mouse melanocytes and mouse melanoma cells, where their levels are directly modulated by the degree of pigmentation. Finally, we identified the precise pigment production pathway controlling the expression of these genes, namely melanocortin 1 receptor (MC1R) signaling. These results suggest that pigment production might underlie the differential expression of angiogenesis-related pathways between Black and White individuals. Based on these findings, we propose that modulation of these genes or their products may be leveraged for precision therapeutics of angiogenesis-dependent diseases characterized by racial disparity.

## Materials and methods

All animal experiments were approved by the Massachusetts General Hospital Institutional Animal Care and Use Committee (IACUC) under protocol 2017N000079. The Boston Children’s Hospital Institutional Review Board has determined that this research qualifies as exempt from the requirements of human subject protection regulations.

### Human RNAseq data analysis

To identify angiogenesis-related genes and pathways that might be regulated by pigmentation in humans, we analyzed RNAseq data from the Genotype-Tissue Expression (GTEx) project, under authorized usage (dbGaP accession phs000424.v7.p2) [12]. Specifically, we focused on samples from Black and White individuals and tissues with angiogenic activity shown to be regulated by melanocyte secretions [10, 11], namely non-sun-exposed skin, tibial artery, and whole blood. First, we used the Short Read Archive (SRA) Toolkit (https://github.com/ncbi/sra-tools) and its fastq-dump utility to fetch all available FASTQ files from the three tissues of interest. S1 Table lists the samples used, including their identifiers, quality control information, and comprehensive individual level data such as race, sex, age, causes of death, and postmortem handling information. The fastq-dump command used was fastq-dump -F—split-files—gzip—tries 10 -O <output_dir> <SRR_ID>. In all, we obtained RNAseq data of 257 non-sun-exposed skin samples from 35 Black and 222 White individuals, 336 tibial artery samples from 50 Black and 286 White individuals, and 815 whole blood from 112 Black and 703 White individuals (S1 Table). We ensured the quality of the data using FastQC [13] version 0.11.6, and quality-trimmed it using Trimmomatic [14] version 0.36 with parameters ILLUMINACLIP:Truseq_adapter_sequence_file.fa:2:30:10:1:true HEADCROP:12 MAXINFO:40:0.7 MINLEN:36. Then, we used STAR version 2.5.3b [15] to align the trimmed FASTQs to the GRCh38.p12 reference human genome, using GENCODE V26 annotations. Specifically, a STAR index was generated using STAR—runThreadN 4—runMode genomeGenerate—genomeDir <genome_dir>—genomeFastaFiles GRCh38.primary_assembly.genome.fa—sjdbGTFfile gencode.v26.primary_assembly.annotation.gtf—sjdbOverhang 88. Then mapping was done using STAR—runThreadN 6—genomeDir <genome_dir>—readFilesIn <trimmed_paired_fastq_1.fq.gz> <trimmed_paired_fastq_2.fq.gz>—readFilesCommand gunzip -c—outFileNamePrefix <SRR_ID>—outReadsUnmapped None—outSAMtype BAM SortedByCoordinate—outSAMmode Full—outFilterMultimapNmax 1—outFilterMismatchNoverLmax 0.05—alignSJoverhangMin 8—alignSJDBoverhangMin 1—outFilterMismatchNmax 999—alignIntronMin 20—alignIntronMax 1000000—alignMatesGapMax 1000000. We then quantified GENCODE V26 Genes using HTSeq-count [16] version 0.11.1 with the following command: htseq-count -f bam -r name -s no -t exon -i gene_id—additional-attr = gene_name -m union—nonunique = all <bam> gencode.v26.primary_assembly.annotation.gtf. Using edgeR version 3.22.5 in R version 3.5.2., we quantified counts per million (CPM) and kept only those genes with at least 1 CPM in at least 100 samples for downstream analyses, for a total of 39,202 out of 58,283 genes. Finally, we normalized the data using trimmed mean of M-values (TMM) normalization [17].

### Differential gene expression analysis

As detailed in S1 Code, we used Limma [18] version 3.36.5 to compare gene expression between samples from Black and White individuals in each of the three tissues, while controlling for age and sex. For that, we first integrated individual level data with the columns of the expression matrix, and created a design matrix based on race, age, and sex. To ensure the comparability of our analyses across tissues, we compared equal proportions of Black and White samples for each tissue. Specifically, for each tissue, we randomly resampled White individuals such that their total count would be exactly three time that of Black individuals, consistent with previous studies [19–21], thereby eliminating differential group size biases. We ran this resampling procedure 100 times and considered the averaged statistics for the differential expression of each gene across all resampled comparisons. Namely, we considered the average expression, average log fold change, average P value, and average adjusted P value across 100 resamples.

### Gene set enrichment analysis (GSEA)

We used GSEA [22] to assess pathway- and mechanism-level differential expression between samples from Black and White individuals in each of the three tissues. For that, MsigDB version 6.2 was used for annotating genes into gene ontology (GO) terms via the following command: java -cp gsea-3.0.jar -Xmx8g xtools.gsea.Gsea -res >expression_matrix> -cls <sample_annotations> -gmx c5.all.v6.2.symbols.gmt -collapse false -mode Max_probe -norm meandiv -nperm 1000 -permute phenotype -rnd_type no_balance -scoring_scheme weighted -rpt_label <analysis_name> -metric Signal2Noise -sort real -order descending -create_gcts false -create_svgs false -include_only_symbols true -make_sets true -median false -num 100 -plot_top_x 50 -rnd_seed timestamp -save_rnd_lists false -set_max 500 -set_min 15 -zip_report false -out <out_dir> -gui false.

### Network level analyses

The STRING database of protein-protein interactions (PPIs) was used for all network level analyses and visualizations [23].

### Graphics

All plots were generated in ggplot2 [24] version 3.3.0, with the exception of heatmaps. Expression heatmaps were created using the heatmap.2 function from the gplots package version 3.1.1.

### Cell culture

Mouse melanocytes, specifically Melan-a cells from black C57BL/6J mice and Melan-e1 cells from white C57BL/6J Mc1r-/- mice [25] (gift from Prof. Dorothy C. Bennett, University of London), were grown in RPMI-1640 medium (Sigma) supplemented with 10% fetal bovine serum (Peak Serum), 1% penicillin-streptomycin (GIBCO), 0.5% 2-mercaptoethanol (GIBCO) and 1% HEPES (GIBCO) at 37°C in a 10% CO_2_-containing environment. The Melan-a cells were supplemented with 200 nnM tetradecanoyl phorbol acetate (TPA) (Sigma), while the Melan-e1 cells were supplemented with 200 nM TPA and 40 pM cholera toxin (Sigma). B16-F1 melanoma cells from black C57BL/6J mice [26] and B16-4GF melanoma cells from white C57BL/6J Mc1r-/- mice (gift from Prof. Hyejung Jung, Ewha Womans University, Seoul, Korea) were grown in DMEM (GIBCO) supplemented with 10% fetal bovine serum and 1% penicillin-streptomycin at 37°C, in a 5% CO_2_-containing environment.

### Total RNA extraction and quantitative real-time PCR (qRT-PCR)

Total RNA was extracted in triplicate using the IBI Isolate Total Extraction Reagent System (IBI Scientific), and cDNA was synthesized using a High Capacity cDNA Reverse Transcription Kit (Applied Biosystems). qRT-PCR was performed to determine relative gene expression in pigmented versus non-pigmented mouse melanocytes using a LightCycler 480 instrument (Roche) with PrimeTime Gene Expression Master Mix (IDT DNA) and the following primers: Apoe–S, TGGAGGCTAAGGACTTGTTTC; Apoe-AS, CACTCGAGCTGATCTGTCAC; Fgfr1–S, GAGCATCAACCACACCTACC; Fgfr1-AS, CCTTACACATGAACTCCACATTG; Vegfa-S, AGAAAGACAGAACAAAGCCAGA; Vegfa-AS, TGGTGACATGGTTAATCGGT; Ppia–S, CAAACACAAACGGTTCCCAG; and Ppia-AS, TTCACCTTCCCAAAGACCAC. Expression levels were measured relative to that of *Ppia*, encoding peptidylprolyl isomerase A. Statistical significance was assessed using t-tests.

### Overall statistical considerations

All P values were corrected for multiple testing using the Benjamini-Hochberg approach [27], ensuring that the false discovery rate (FDR) of this study is below 0.05.

## Results

### Angiogenesis pathways are differentially expressed between Black and White individuals

We first sought to identify genes and pathways that are robustly differentially expressed between Black and White individuals in tissues with angiogenic activity shown to be regulated by melanocyte secretions [10, 11]. Toward this goal, we leveraged large-scale RNAseq data of the GTEx project, specifically that from skin that had not been sun-exposed, tibial artery, and whole blood (S1 Table). While maintaining a ratio of 1:3 between Black and White samples across tissues and controlling for FDR at 5% (see Methods), we detected 1,653 differentially expressed genes (DEGs) in non-sun-exposed skin (Fig 1, S2 and S3 Tables), 1,462 DEGs in the tibial artery (Fig 2, S2 and S4 Tables), and 748 DEGs in whole blood (Fig 3, S2 and S5 Tables). Of these, 67 genes were differentially expressed between Black and White individuals in all three tissues, 258 were differentially expressed in two tissues, and the rest were tissue-specific DEGs (Fig 4 and S2 Table).

**Fig 1:** DEGs between Black and White individuals in non-sun-exposed skin. (A) Expression heatmap of the top 100 DEGs in 257 non-sun-exposed skin tissue samples, showing the result of a two-way unsupervised hierarchical clustering. Each row represents a DEG and each column represents a sample. The order of genes and samples was determined in an unsupervised manner, based on similarities in expression profiles, and is detailed in S3 Table. Samples are color coded according to their reported race. Expression values are presented in log(TMM), scaled according to the color key in the top left corner. (B) Volcano plot depicting the magnitude and significance of expression differences at the single gene level. For each gene expressed in non-sun-exposed skin, the log_2_ fold change of normalized expression between Black and White individuals is shown on the X axis, and the negative log_10_ of its FDR-adjusted P value is shown on the Y axis. Positive X values represent upregulation in Black individuals and negative X values represent downregulation. Significant DEGs are in red and the symbols of the 10 most significant ones are noted. DEG, differentially expressed gene.

**Fig 2:** DEGs between Black and White individuals in the tibial artery. (A) Expression heatmap of the top 100 DEGs in 336 tibial artery tissue samples, showing the result of a two-way unsupervised hierarchical clustering. Each row represents a DEG and each column represents a sample. The order of genes and samples was determined in an unsupervised manner, based on similarities in expression profiles, and is detailed in S4 Table. Samples are color coded according to their reported race. Expression values are presented in log(TMM), scaled according to the color key in the top left corner. (B) Volcano plot depicting the magnitude and significance of expression differences at the single gene level. For each gene expressed in the tibial artery, the log_2_ fold change of normalized expression between Black and White individuals is shown on the X axis, and the negative log_10_ of its FDR-adjusted P value is shown on the Y axis. Positive X values represent upregulation in Black individuals and negative X values represent downregulation. Significant DEGs are in red and the symbols of the 10 most significant ones are noted. DEG, differentially expressed gene.

**Fig 3:** DEGs between Black and White individuals in whole blood. (A) Expression heatmap of the top 100 DEGs in 815 whole blood samples, showing the result of a two-way unsupervised hierarchical clustering. Each row represents a DEG and each column represents a sample. The order of genes and samples was determined in an unsupervised manner, based on similarities in expression profiles, and is detailed in S5 Table. Samples are color coded according to their reported race. Expression values are presented in log(TMM), scaled according to the color key in the top left corner. (B) Volcano plot depicting the magnitude and significance of expression differences at the single gene level. For each gene expressed in whole blood, the log_2_ fold change of normalized expression between Black and White individuals is shown on the X axis, and the negative log_10_ of its FDR-adjusted P value is shown on the Y axis. Positive X values represent upregulation in Black individuals and negative X values represent downregulation. Significant DEGs are in red and the symbols of the 10 most significant ones are noted. DEG, differentially expressed gene.

**Fig 4:** Venn diagram of DEGs across tissues. Overlapping regions represent DEGs shared between comparisons. The color scale is proportional to the number of DEGs.

Gene set enrichment analysis was next used to identify gene expression differences between White and Black individuals at the whole pathway level. Several angiogenesis pathways were found to be up-regulated in White individuals, including artery morphogenesis (Normalized Enrichment Score (NES) = 2.07, P = 2.10 x 10^−3^), regulation of endothelial cell chemotaxis (NES = 2.03, P = 3.99 x 10^−3^), and cellular response to vascular endothelial growth factor stimulus (NES = 2.03, P = 7.91 x 10^−3^, Fig 5A). These findings are consistent with the observed elevated burden of angiogenesis-dependent diseases in White, as compared to Black individuals [1–3].

**Fig 5:** Angiogenesis pathways differentially expressed between Black and White individuals and the network structure of interactions between their leading-edge gene products. (A) Convergence of DEGs between Black and White individuals on angiogenic functions. Shown are enriched Gene Ontology (GO) annotations among DEGs between Black and White individuals, as measured in whole blood RNAseq. (B-D) Relationships between the protein products of genes driving the up-regulation of (B) artery morphogenesis, (C) regulation of endothelial cell chemotaxis, and (D) cellular response to VEGF stimulus in Black, as compared to White individuals. Shown is the PPI network structure of products of leading-edge genes, namely those driving pathway-level differential expression between Black and White individuals. Nodes represent proteins, while their interactions are denoted by color-coded edges: Magenta, experimentally determined interactions; cyan, manually curated interactions; green, interactions reported in PubMed abstracts; black, co-expression; and blue, protein homology. VEGFA, APOE, and FGFR1 are highlighted by a bold black circle because of their network centrality and implication in diseases of racial disparity.

Subsequent network analyses identified several hub genes driving the differential expression of these pathways (Fig 5B–5D). For example, leading-edge genes (i.e. whose expression correlates most with skin color) of the artery morphogenesis pathway, whose protein products are most central to the PPI network of this pathway, include those encoding vascular endothelial growth factor A (VEGFA), platelet-derived growth factor receptor beta (PDGFRB), Jagged-1 (JAG1), Notch receptor 3 (NOTCH3), and Hes family BHLH transcription factor 1 (HES1). Notably, apolipoprotein E (APOE), which is directly connected to the products of three other members of this network, is known for its anti-angiogenic functions [28] and has been implicated in several diseases with racial disparity, including Alzheimer’s disease [29] and age-related hearing loss [30] (Fig 5B). Similarly, Fig 5C depicts the PPI network of leading-edge gene products involved in endothelial cell chemotaxis, highlighting the centrality of VEGFA. One notable member of this network is fibroblast growth factor receptor 1 (FGFR1), which was shown to be a key driver of melanoma angiogenesis and treatment resistance [31], common phenomena in Black individuals [32]. Finally, interactions between the protein products of leading-edge genes of the cellular response to the VEGF stimulus pathway are shown in Fig 5D.

### *VEGFA*, *APOE*, and *FGFR1* are differentially expressed between Black and White individuals

We next focused on the expression of genes driving the observed pathway-level differential expression between Black and White individuals, specifically those genes whose protein products are central to the PPI network of these pathways (designated by bold circles in Fig 5B–5D). We found that *VEGFA* expression is down-regulated in Black, as compared to White individuals (log_2_ fold-change (logFC) = -0.57, P = 6.06 x 10^−5^, FDR-adjusted P = 3.50 x 10^−3^, Fig 6A), while *APOE* and *FGFR1* are up-regulated in Black, as compared to White individuals (*APOE* logFC = 1.19, P = 5.17 x 10^−8^, FDR-adjusted P = 2.18 x 10^−5^, Fig 6B; *FGFR1* logFC = 0.44, P = 1.56 x 10^−3^, FDR-adjusted P = 3.29 x 10^−2^; Fig 6C). To test whether the expression of these genes directly depends on pigmentation levels, we next considered two cellular systems of melanocortin 1 receptor (MC1R) signaling, a major determinant of human pigmentation.

**Fig 6:** Differential expression of *VEGFA*, *APOE*, and *FGFR1* between Black and White individuals. (A) Down-regulation of *VEGFA* expression in whole blood from Black, as compared to White individuals. (B) Up-regulation of arterial *APOE* expression in Black, as compared to White individuals. (C) Up-regulation of *FGFR1* expression in non-sun-exposed skin from Black, as compared to White individuals.

### *Vegfa*, *Apoe*, and *Fgfr1* expression is pigmentation-dependent and controlled by melanocortin 1 receptor (Mc1r) signaling

MC1R is a key regulator of pigment production, whose genomic variants are largely responsible for pigmentation differences in humans [33]. Therefore, we used two cellular systems of murine MC1R function to examine the impact of pigmentation on *Vegfa*, *Apoe*, and *Fgfr1* expression. The first is an isogenic system of *MC1R* loss-of-function in mouse melanocytes [25], while the second is an isogenic system of *MC1R* loss-of-function in the mouse B16 melanoma cell line [34]. Each system allows for analysis of the direct effect of MC1R function, and thereby pigment production, on gene expression in an isogenic background. Using these two systems, we demonstrated that the expression of *Vegfa*, *Apoe*, and *Fgfr1*, which drive the differential expression of angiogenesis pathways between White and Black individuals, depends on pigment production via MC1R. Specifically, we found that *Vegfa* gene expression is 1.56-fold up-regulated in non-pigmented, as compared to pigmented mouse melanocytes (Student’s t-test P = 6.58 x 10^−3^), and 5.12-fold up-regulated in non-pigmented, relative to pigmented, mouse melanoma cells (Student’s t-test P = 1.43 x 10^−6^, Fig 7A). Moreover, *Apoe* levels were 235.56-fold up-regulated in pigmented mouse melanocytes, as compared to their non-pigmented counterparts (Student’s t-test P = 8.61 x 10^−3^), and 5.05-fold up-regulated in pigmented versus non-pigmented mouse melanoma cells (Student’s t-test P = 1.79 x 10^−2^; Fig 7B). Similarly, *Fgfr1* levels were 4.5-fold up-regulated in pigmented versus non-pigmented mouse melanocytes (Student’s t-test P = 1.32 x 10^−2^), and 111.6-fold up-regulated in pigmented mouse melanoma cells, relative to non-pigmented such cells (Student’s t-test P = 1.47 x 10^−2^; Fig 7C). These results suggest that the differential expression of angiogenesis pathways between Black and White individuals depends on pigmentation levels and is regulated by MC1R signaling. Moreover, these results demonstrate that out of the heterogenous cell populations that comprise the bulk RNAseq data and that could have contributed to the observed expression measurements, melanocytes *per se* express *VEGFA*, *APOE*, and *FGFR1*. This experiment also showed that melanocytes *per se* express factors that regulate the expression of these genes, and that these regulatory factors depend on MC1R signaling.

**Fig 7:** MC1R-dependent expression of *Vegfa*, *Apoe*, and *Fgfr1*. Two isogenic cellular systems of MC1R loss-of-function were used to define relationships between pigmentation and the expression of (A) *Vegfa*, (B) *Apoe*, and (C) *Fgfr1*. Consistent with findings in Black and White individuals shown in Fig 6, *Vegfa* was found to be down-regulated in pigmented, as compared to non-pigmented cells, while *Apoe* and *Fgfr1* were both up-regulated in pigmented versus non-pigmented cells.

## Discussion

This study identified angiogenesis-related genes and pathways that are differentially expressed between Black and White individuals. It was specifically shown that the expression of *VEGFA*, *APOE*, and *FGFR1* –central angiogenesis-related pathway genes–depends on MC1R signaling and is thereby directly modulated by pigmentation levels. As such, this study improves our understanding of the impact of pigmentation on angiogenesis, and moves us one step closer toward precision medicine of angiogenesis-dependent diseases characterized by racial disparity.

Melanogenesis, the complex process by which melanocytes produce melanin, is stimulated by several factors, including ultraviolet (UV) irradiation, melanocyte-stimulating hormone (MSH), fibroblast growth factor 2 (FGF2), and the tyrosinase-catalyzed oxidation of tyrosine. Upon UV irradiation, α-MSH secreted by keratinocytes binds to MC1R, a G protein-coupled receptor expressed on the melanocyte surface that serves as a key regulator of pigment production. In mouse models and human studies, polymorphisms in *MC1R* have been associated with the levels and types of melanin produced [35–37]. The present study suggests that MC1R function controls the expression of angiogenesis pathways by directly modulating the expression of their driver genes.

Differences in angiogenesis gene expression between Black and White individuals could be advantageous in some conditions and deleterious in others. For example, angiogenesis should be blocked in AMD and infantile hemangioma. However, in cutaneous lupus erythematosus and wound healing, angiogenesis should be enhanced. Therefore, any potential modulation of pigment-mediated angiogenesis gene expression to minimize racial disparities should be condition-specific.

Consistent with the present results showing up-regulation of angiogenesis pathways in White, as compared to Black individuals, we have previously shown that non-pigmented melanocytes promote angiogenesis *in vitro* and *in vivo*, and that FMOD contributes to this effect [11]. The present study thus expands our understanding of the molecular links between pigmentation levels and angiogenesis, and offers further avenues for closing the racial disparity gap in angiogenesis-dependent diseases.

## Supporting information

S1 Table Detailed sample information. (XLSX)

S2 Table DEGs between Black and White individuals in tissues with angiogenic activity. (XLSX)

S3 Table Genes and samples in Fig 1A. The top 100 DEGs in 257 non-skin-exposed skin samples from Black as compared to White individuals, ordered according to two-way hierarchical clustering.
(XLSX)

S4 Table Genes and samples in Fig 2A. The top 100 DEGs in 336 tibial artery samples from Black as compared to White individuals, ordered according to two-way hierarchical clustering.
(XLSX)

S5 Table Genes and samples in Fig 3A. The top 100 DEGs in 815 whole blood samples from Black as compared to White individuals, ordered according to two-way hierarchical clustering.
(XLSX)

S1 Code (R)
